The article "The High Expression of Adhering and Circulating Integrin Serves as a Diagnostic Marker in Venous Thromboembolism" was retracted in 2023. Reasons: signs of a paper mill; compromised peer review; unreliable results or conclusions.

# The High Expression of Adhering and Circulating Integrin Serves as a Diagnostic Marker in Venous Thromboembolism

**DOI:** 10.1155/2022/9610071

**Published:** 2022-10-07

**Authors:** Fan Yang, Yanli Song, Haoming Song, Weiping Zheng, Lemin Wang

**Affiliations:** ^1^Department of Clinical Laboratory, Tongji Hospital, Tongji University School of Medicine, Shanghai, 200065, China; ^2^Department of Internal Emergency, Tongji Hospital, Tongji University School of Medicine, Shanghai, 20006, China; ^3^Department of Cardiology, Tongji Hospital, Tongji University School of Medicine, Shanghai, 200065, China

## Abstract

**Objective:**

To investigate the diagnostic value of circulating integrins *β*1, 2, and 3 in venous thrombosis (VTE).

**Materials and Methods:**

A total of 474 VTE patients and 306 patients with nonhigh risk for VTE as the control group were studied. Levels of adhering integrins *β*1, 2, and 3 were detected by flow cytometry. Levels of circulating integrins *β*1, 2, and 3 in serum were measured by enzyme-linked immunosorbent assay.

**Results:**

We found that integrins *β*1, 2, and 3 were expressed highly both in serum and on the surface of leukocytes and platelets in venous thromboembolism. The levels of circulating integrins *β*1, 2, and 3 are positively correlated with adhering integrins. It showed excellent clinical diagnostic performance of circulating integrins *β*1, 2, and 3 in venous thromboembolism.

**Conclusions:**

Integrin subunit *β* can be used as a diagnostic marker with high sensitivity and specificity for venous thromboembolism.

## 1. Introduction

Venous thromboembolism (VTE) includes deep venous thrombosis (DVT) and pulmonary thromboembolism (PE). Acute pulmonary embolism is the third most common cause of cardiovascular mortality, with high mortality rates [1]. And there are many misdiagnoses or missed diagnosis in deep venous thrombosis [2]. Making a rapid and definite diagnosis followed by immediate and appropriate therapy may help to improve this severe situation. Now, VTE can be diagnosed mostly by imaging technique such as color Doppler ultrasound of deep vein or pulmonary angiography, instead of experimental marker [3]. D-dimer is a commonly used marker, but it is mostly used as an excluding index rather than a diagnostic marker [4, 5]. So it is urgent and significant to find a new marker for early diagnosis in VTE.

In previous study, acute venous thrombus was analyzed by tandem mass spectrometry. It is found that integrin *β* molecules are the core proteins of the thrombus protein network by bioinformatic analysis [6]. The mRNA level of integrins *β*1, *β*2, and *β*3 was significantly upregulated in symptomatic VTE [7]. Integrin *β*1 was localized on the surface of lymphocytes, integrin *β*2 was localized on the surface of leukocytes, and integrin *β*3 was localized on the surface of platelets in venous thrombus by immunohistochemistry [8]. According to previous results, integrin *β* molecule may be a new marker for early diagnosis in VTE.

In this study, a multicentric research is developed by 5 hospitals (Tongji Hospital belongs to Tongji University, Shanghai, East of China; Fuwai Hospital belongs to Chinese Academy of Medical Sciences, Beijing, North of China; Tongji Hospital belongs to Tongji Medical College, Huazhong University of Science & Technology, Wuhan, Middle of China; First Affiliated Hospital belongs to Xian JiaoTong University, Xian, West of China; and Affiliated Hospital belongs to Guangdong Medical University, Xian, South of China). We collected 474 cases of acute venous thrombus which were diagnosed by color Doppler ultrasound of the deep vein or pulmonary angiography. We also collected 306 cases of patients with no high risk factors for VTE as the control group. Flow cytometry was used to examine the levels of integrins *β*1, *β*2, and *β*3 expressed on the surface of leucocyte, lymphocyte, and platelet in all these patients. Enzyme-linked immunosorbent assay (ELISA) was performed to detect the levels of circulating integrins *β*1, *β*2, and *β*3 in serum in all these patients. We analyzed diagnostic performance of integrin subunit *β* as a marker for early diagnosis of VTE.

## 2. Materials and Methods

The subjects included patients with a definite diagnosis between March, 2011, and May, 2015, in 5 hospitals above. The methods and steps of detection were based on the technical manual of the reagent manufacturer, and the results were analyzed by statistic software. The detection did not influence the treatment of all patients.

### 2.1. Study Population

A total of 474 VTE patients (256 males and 218 females, mean age = 62.46 ± 13.12) were enrolled from 5 hospitals. In VTE patients having DVT and/or PE, the diagnosis was confirmed by color Doppler ultrasound of the deep vein or pulmonary angiography. The control group (306 patients) consisted of patients with non-risk factor, and patients with VTE, acute infection, cancer, autoimmune diseases, trauma, and recent surgical treatment were excluded.

### 2.2. Methods for Detection

(1) Levels of adhering integrins *β*1, *β*2, and *β*3 expressed on surface of cell membrane were detected by EPICS XL-4 flow cytometry (Beckman Coulter) and analyzed using System II software. Fluorescent antibodies of integrin *β*1 (CD29, PE dye), integrin *β*2 (CD18, PE dye), and integrin *β*3 (CD61, PE dye) were provided by Invitrogen Company. Hemolytic reagent was provided by BD Company
  - We collected 2 ml peripheral blood from the patients with EDTA anticoagulated both in VTE patients and in the control group. FACS must be done in 2 h after collection of samples
  - 100 *μ*l EDTA anticoagulated peripheral blood was added to each tube for detecting integrins *β*1, *β*2, and *β*3 separately. Isotype control was also added into each tube. Integrin *β*1 and integrin *β*2 were mixed with 20 *μ*l mouse IgG1-PE, and integrin *β*3 was mixed with 20 *μ*l mouse IgG2-PE. Then, 20 *μ*l fluorescent antibody (CD29, CD18, and CD61) was added to each tube. After mixing for 30 sec, each tube was incubated at room temperature keeping out of light for 30 min. After that, 500 *μ*l hemolysin was added in teach tube and mixed for 30 sec; then, each tube was incubated at 37°C keeping out of light for 30 min and washed by phosphoric acid buffer at least 3 times; 500 *μ*l sheath fluid was added and then detected by flow cytometry
  - The standardized Beckman-Coulter fluorescent microspheres were used to adjust the PMT voltage, fluorescence compensation, and sensitivity. At least 10000 cells were collected in the experiment. The scattered plot of isotype control was used for gating at corresponding cells. Integrin *β*1 and integrin *β*2 gating was lymphocytes, and integrin *β*3 gating was platelets. According to the fluorescence intensity in four-quadrant diagrams, the percentage of positive cells in all counting cells was calculated. Data were analyzed with System II software automatically
(2) Levels of circulating integrins *β*1, *β*2, and *β*3 expressed in serum were detected by Human Integrin Beta-1, 2, and 3. ELISA kits were provided by CUSABIO Company
  - We collected 2 ml peripheral blood from the patients with EDTA anticoagulated both in VTE patients and in the control group. Then, using a serum separator tube, samples are allowed to clot for 2 h at room temperature or overnight at 4°C before centrifugation for 15 m at 1000∗g. Remove serum and assay immediately or aliquot, and store samples at -20°C or -80°C. Avoid repeated freeze-thaw cycles
  - Adding 25 *μ*l serum samples to 225 *μ*l of sample diluent to induce 10-fold dilution
  - Reconstitute the standard with 1.0 ml of sample diluent. This reconstitution produces a stock solution. Use the stock solution to produce a 2-fold series to make a standard curve
  - Add 100 *μ*l of standard and sample per well. Incubate for 2 h at 37°C. Then, add 100 *μ*l of biotin antibody to each well. Incubate for 1 h at 37°C. Wash with wash buffer for 3 times. Add 100 *μ*l of HRP-avidin to each well. Incubate for 1 h at 37°C. Wash 3 times. Add 90 *μ*l of TMB substrate to each well. Incubate for 15-30 m at 37°C. Add 50 *μ*l of Stop Solution to each well
  - Determine the optical density of each well within 5 m, using a microplate reader (ELx-800, BIOTEK) set to 450 nm (wavelength correction set to 540 nm). Create a standard curve by reducing the data using computer software capable of generating a four-parameter logistic (4-PL) curve fit. The data may be linearized by plotting the log of the Integrin Beta-1, 2, and 3 concentrations versus the log of the O.D., and the best fit line can be determined by regression analysis

## 3. Statistical Analysis

All the results are expressed as means ± SD or medians. To compare clinical data between groups, we used Student's *t* test or Wilcoxon signed rank test as appropriate. Pearson correlation analysis was used to compare circulating integrin subunits *β*1, *β*2, and *β*3 in serum with adhering integrin on the surface of leukocytes and platelets. Receiver operating characteristic curve was used to analyze the clinical diagnostic performance of circulating integrin subunits *β*1, *β*2, and *β*3 in venous thrombosis.

SPSS 18.0 software was used for statistical analysis. Statistical significance was defined as *P* < 0.05.

## 4. Results

A total of 474 patients of VTE were including 54.01% males and 45.99% females, with a mean age of 62.46 ± 13.12 years, while control group of patients were including 52.94% males and 47.06% females, with a mean age of 56.85.46 ± 16.24 years. Levels of adhering integrins and circulating integrins were detected in these patients.

Adhering integrins *β*1 (CD29), *β*2 (CD18), and *β*3 (CD61) were highly expressed in VTE patients which was determined by flow cytometry as shown in Figure 1. The median levels of adhering integrin *β*1 in VTE patients (14.5 ± 7.19%) were higher than those in the control group patients (8.52 ± 2.69%) (*P* < 0.001), adhering integrin *β*2 in VTE patients (94.01 ± 5.85%) was higher than that in the control group patients (87.42 ± 6.45%) (*P* < 0.001), and adhering integrin *β*3 in VTE patients (11.87 ± 4.3%) was higher than that in the control group patients (9.55 ± 2.59%) (*P* < 0.001) as shown in Figure 2.

Circulating integrins *β*1, *β*2, and *β*3 were determined by enzyme-linked immunosorbent assay. The median levels of circulating integrin *β*1 in VTE patients (2213.11 ± 1089.07 pg/ml) were higher than those in the control group patients (1233.47 ± 397.65 pg/ml) (*P* < 0.001), circulating integrin *β*2 in VTE patients 160.18 ± 65.33 pg/ml) was higher than that in the control group patients (102.93 ± 42.45 pg/ml) (*P* < 0.001), and circulating integrin *β*3 in VTE patients (237.54 ± 90.28 pg/ml) was higher than that in the control group patients (155.6 ± 47.18 pg/ml) (*P* < 0.001) as shown in Figure 3.

When a comparison was made between circulating integrins and adhering integrins in VTE patients, we found that circulating integrins *β*1, *β*2, and *β*3 were highly positively correlated with adhering integrins *β*1, *β*2, and *β*3, respectively (*P* = 0.024, 0.027, and 0.032,) as shown in Table 1.

ROC curve analysis was used to assess diagnostic performance of circulating integrins *β*1, *β*2, and *β*3. When a comparison was made between VTE patients and non-VTE patients, the AUC of integrin *β*1 was 0.817 (95% CI: 0.789-0.846, *P* < 0.001), the AUC of circulating integrin *β*2 was 0.813 (95% CI: 0.782-0.843, *P* < 0.001), and the AUC of circulating integrin *β*3 was 0.837 (95% CI: 0.810-0.864, *P* < 0.001,) as shown in Figure 4 and Table 2. According to the ROC curve, the diagnostic performance of circulating integrins *β*1, *β*2, and *β*3 was assessed as shown in Table 2. The optimum cutoff of circulating integrins *β*1, *β*2, and *β*3 was 1374 pg/ml, 128.5 pg/ml, and 184.5 pg/ml, respectively.

ROC curve analysis was also used to assess diagnostic performance of combination of circulating integrins *β*1, *β*2, and *β*3. When a comparison was made between VTE patients and non-VTE patients, binary logistic regression analysis was made as shown in Tables 3; the logistic regression equation was logit(*P*) = −12.756 + 0.002 integrin *β*1 + 0.034 integrin *β*2 + 0.028 integrin *β*3. Then, the ROC curve of a combination with circulating integrins *β*1, *β*2, and *β*3 was made and the AUC was 0.951 (95% CI: 0.937-0.965, *P* < 0.001) as shown in Figure 5 and Table 4. According to the ROC curve, the diagnostic performance of the combination of circulating integrins *β*1, *β*2, and *β*3 was assessed as shown in Table 4.

## 5. Discussion

Venous thromboembolism is a severe disease which is often misdiagnosed or has missed diagnosis. One important reason is lacking experimental marker. D-dimer is wildly used as diagnostic marker, but it is more valuable as an excluding index [5]. Integrin *β* molecules are the core proteins of the thrombus protein network and may be a new marker for early diagnosis in VTE. So we performed this study for large samples of VTE patients collected from 5 hospitals in different regions in China.

In this study, we found that the levels of integrins *β*1 and *β*2 in the VTE group were significantly higher than in those in the control group expressed on the surface of lymphocytes. We also found that the levels of integrin *β*3 in the VTE group were significantly higher than those in the control group expressed on the surface of platelets. Integrins are cell adhesion receptors; they play an important role in the interaction between cells and extracellular matrix and cell and cell interactions by combining with its ligands. Integrins are heterodimers consisting of *α* and *β* subunits. They consist of at least 18 *α* and 8 *β* subunits, producing 24 different heterodimers [9]. The main function of *β* subunits is to transfer activating message between intracellular and extracellular [10]. Therefore, the high expression of integrin *β*1 level indicates the activation of lymphocytes, which is correlated with inflammation, thrombosis, and tumor after integrating with its ligands including laminins, collagens, thrombospondin, vascular cell adhesion molecule 1, and fibronectin. The high expression of integrin *β*2 level indicates the activation of white cells, which is correlated with inflammation and thrombosis after integrating with its ligands including fibrinogen, complement component iC3b, intracellular adhesion molecule-1, and factor X. The high expression of integrin *β*3 level indicates the activation of platelets, which is correlated with platelet aggregation and thrombus after integrating with its ligands including fibrinogen, fibronectin, vitronectin, von Willebrand factor (vWF), and thrombospondin [11–13].

Integrins will fall off from the surface of cell membrane and turn into circulating form in peripheral blood which can be tested in serum. In our study, circulating integrins *β*1, *β*2, and *β*3 expressed in the VTE group were also obviously higher than those in the control group. Moreover, we found that the level of circulating integrins *β*1, *β*2, and *β*3 was positively correlated with the level of adhering integrin (correlation coefficients 0.609, 0564, and 0.658, respectively). The findings reported here may have major clinical implications. We believed that circulating integrins *β*1, *β*2, and *β*3 expressed in serum may be a likely possible diagnostic marker for VTE due to the lack of detection standard of adhering integrin. Furthermore, quantitative method of ELISA for detecting circulating integrins in serum is more convenient and faster than semiquantitative method of FACS. To our knowledge, no previous study has reported that circulating integrins *β*1, *β*2, and *β*3 can be used as a marker for early diagnosis in VTE. In our study, it is shown there that some patients who were diagnosed as having venous thrombosis definitely did not express integrins *β*1, *β*2, and *β*3 highly. Contrarily, there are some patients in the control group who had upgraded expression of integrins *β*1, *β*2, and *β*3. We do not have a precise explanation for this situation.

By the ROC curve, we found that circulating integrins *β*1, *β*2, and *β*3 have great sensitivity and specificity. The AUC of circulating integrins *β*1, 2, and 3 were 0.817, 0.813, and 0.837. The optimum cutoff of circulating integrins *β*1, *β*2, and *β*3 was 1374 pg/ml, 128.5 pg/ml, and 184.5 pg/ml, respectively. When combined with circulating integrins *β*1, *β*2, and *β*3, the AUC was upgraded to 0.951, and sensitivity and specificity were improved to 85.9% and 90.5%, while for D-dimer, it was reported that the AUC was 0.811 [14]. D-dimer is the most common index used in the diagnosis of VTE. The negative value of D-dimer may safely rule out both DVT and PE with a high sensitivity of 83%-96% and a negative predictive value of nearly 100%. However, due to its low specificity (around 40%), D-dimer is not a perfect diagnostic index for VTE [15–18]. It showed that the combination of circulating integrins *β*1, *β*2, and *β*3 has better diagnostic performance than D-dimer in VTE. If we determined both circulating integrins and D-dimer, there may be more diagnostic efficiency in VTE.

In conclusion, integrin *β* molecules are core proteins of venous thrombi. And circulating integrins *β*1, *β*2, and *β*3 have high specificity and sensitivity in the diagnosis of VTE; these proteins may be a possible diagnostic marker. If determining both D-dimer and integrins, venous thromboembolism may be diagnosed in the early stage before imaging changes. However, our findings require further confirmation by studies with a larger cohort.

## Figures and Tables

**Figure 1:** (a) Integrin *β*1 (CD29) levels expressed on the surface of lymphocytes; (b) integrin *β*2 (CD18) levels expressed on the surface of lymphocytes; (c) integrin *β*3 (CD61) levels expressed on the surface of platelets, which were determined by flow cytometry.

**Figure 2:** The median levels of adhering integrins *β*1, *β*2, and *β*3 were all significantly higher in VTE patients when compared with control group patients (*P* < 0.001, *P* < 0.001, and *P* < 0.001, respectively).

**Figure 3:** The median levels of circulating integrins *β*1, *β*2, and *β*3 were all significantly higher in VTE patients when compared with control group patients (*P* < 0.001, *P* < 0.001, and *P* < 0.001, respectively).

**Figure 4:** Receiver operating characteristic (ROC) curves for assessing the diagnostic performance of circulating integrins *β*1, *β*2, and *β*3 in VTE patients. The area under the curve (AUC) of circulating integrin *β*1 was 0.817 (*P* < 0.001), AUC of circulating integrin *β*2 was 0.813 (*P* < 0.001), and AUC of circulating integrin *β*3 was 0.837 (*P* < 0.001).

**Figure 5:** Receiver operating characteristic (ROC) curves for assessing the diagnostic performance of the combination of circulating integrins *β*1, *β*2, and *β*3 in VTE patients. The area under the curve (AUC) of the combination of integrins was 0.951 (*P* < 0.001).

**Table 1:** Correlation between circulating integrins *β*1, *β*2, and *β*3 and adhering integrins *β*1, *β*2, and *β*3.

	Circulating integrin *β*1	Circulating integrin *β*2	Circulating integrin *β*3
Correlation coefficient	0.609	0.564	0.658
*P* value	0.024	0.027	0.032

**Table 2:** Diagnostic performance of circulating integrins *β*1, *β*2, and *β*3 for VTE.

	Circulating integrin *β*1	Circulating integrin *β*2	Circulating integrin *β*3
AUC	0.817	0.813	0.837
95% confidence interval	0.789-0.846	0.782-0.843	0.810-0.864
Optimum cutoff (pg/ml)	1374	128.5	184.5
Sensitivity	80.4%	76.6%	72.8%
Specificity	82.1%	77.3%	74.2%

AUC: area under the curve.

**Table 3:** Binary logistic regression analysis of circulating integrins for VTE.

	*B*	S.E.	Wald	df	Sig	Exp(*B*)
Integrin *β*1	0.002	0.000	68.044	1	<0.001	1.002
Integrin *β*2	0.034	0.004	82.132	1	<0.001	1.034
Integrin *β*3	0.028	0.003	83.887	1	<0.001	1.028
Constant	-12.756	0.968	173.788	1	<0.001	0.000

**Table 4:** Diagnostic performance of combination of circulating integrins *β*1, *β*2, and *β*3 for VTE.

	Combination of circulating integrins *β*1, *β*2, and *β*3
AUC	0.951
95% confidence interval	0.937-0.965
Sensitivity	85.9%
Specificity	90.5%

AUC: area under the curve.

## Data Availability

All data generated or analyzed during this study are included in this published article.
